RETRACTED

# The prevalence of electronic cigarettes vaping globally: a systematic review and meta-analysis

**DOI:** 10.1186/s13690-022-00998-w

**Published:** 2022-11-21

**Authors:** Hadi Tehrani, Abdolhalim Rajabi, Mousa Ghelichi- Ghojogh, Mahbobeh Nejatian, Alireza Jafari

**Affiliations:** 1 Social Determinants of Health Research Center, Mashhad University of Medical Sciences, Mashhad, Iran; 2 Department of Health Education and Health Promotion, School of Health, Mashhad University of Medical Sciences, Mashhad, Iran; 3 Environmental Health Research Center, Department of Biostatistics and Epidemiology, Faculty of Health, Golestan University of Medical Sciences, Gorgan, Iran; 4 Metabolic Disorders Research Center, Golestan University of Medical Sciences, Gorgan, Iran; 5 Social Determinants of Health Research Center, Gonabad University of Medical Sciences, Gonabad, Iran; 6 Department of Health Education and Health Promotion, School of Health, Social Development and Health Promotion Research Center, Gonabad University of Medical Sciences, Gonabad, Iran

**Keywords:** Electronic cigarette, Vaping, Tobacco, Electronic nicotine, Global

## Abstract

**Background:**

The purpose of this systematic review study was to determine the national, regional, and global prevalence of electronic cigarettes (e-cigarettes) vaping.

**Method:**

The articles were searched in July 2020 without a time limit in Web of Science (ISI), Scopus, PubMed, and Ovid-MEDLINE. At first, the titles and abstracts of the articles were reviewed, and if they were appropriate, they entered the second stage of screening. In the second stage, the whole articles were reviewed and articles that met the inclusion criteria were selected. In this study, search, selection of studies, qualitative evaluation, and data extraction were performed by two authors independently, and any disagreement between the two authors was reviewed and corrected by a third author.

**Results:**

In this study, the lifetime and current prevalence of e-cigarettes vaping globally were 23% and 11%, respectively. Lifetime and current prevalence of e-cigarettes vaping in women were 16% and 8%, respectively. Also, lifetime and current prevalence of e-cigarettes vaping in men were 22% and 12%, respectively. In this study, the current prevalence of e-cigarettes vaping in who had lifetime smoked conventional cigarette was 39%, and in current smokers was 43%. The lifetime prevalence of e-cigarettes vaping in the Continents of America, Europe, Asia, and Oceania were 24%, 26%, 16%, and 25%, respectively. The current prevalence of e-cigarettes vaping in the Continents of America, Europe, Asia, and Oceania were 10%, 14%, 11%, and 6%, respectively.

RETRACTED

**Conclusions:**

Based on the results of this study, it can be concluded that the popularity of e-cigarettes is increasing globally. Therefore, it is necessary for countries to have more control over the consumption and distribution of e-cigarettes, as well as to formulate the laws prohibiting about the e-cigarettes vaping in public places. There is also a need to design and conduct information campaigns to increase community awareness about e-cigarettes vaping.

**Supplementary Information:**

The online version contains supplementary material available at 10.1186/s13690-022-00998-w.

## Background

Electronic cigarettes (e-cigarettes) are another type of tobacco that has become popular in the world in recent years. These cigarettes have batteries and heat the liquid and usually contain nicotine and other toxins [1]. In recent years, the prevalence of e-cigarettes has increased.

The results of a study by Brożek and et al. in several European countries showed that the overall prevalence of lifetime e-cigarette vaping was 43.7%, with 51.3% in men and 40.5% in women [2]. According to the results of various studies, the prevalence of e-cigarettes vaping in different countries such as France, Mexico, China, Australia, and in the United States were 25.46%, 42.42%, 24.44%, 12.52%, and 13.47%, respectively [3–7].

A systematic review by Pisinger and Dossing in 2014 showed that e-cigarettes can have an adverse effect on the health of individuals due to materials such as fine/ultrafine particles, volatile organic compounds, carcinogenic carbonyls, carcinogenic tobacco-specific nitrosamines, and cytotoxicity. Additionally, another major concern is the availability of novel compounds, such as propylene glycol, which are not found in conventional cigarettes with unknown impact on health [8]. The results of studies showed that using e-cigarettes may increase the risk of cardiovascular disease and respiratory disease [9, 10].

People usually e-cigarettes vaping to quit conventional cigarettes, while some people using both types of cigarettes and are at higher risk [11]. The e-cigarettes vaping can also encourage people to initial use of conventional cigarettes and other substances [12, 13]. The results of a systematic review study have shown that adolescents whose parents and friends vaping of e-cigarettes are more likely to be inclined towards e-cigarettes vaping in the future [14]. Therefore, this systematic and meta-analysis review study was conducted with the aims of (1) Investigating an updated estimate of the prevalence of lifetime and current e-cigarettes vaping in around the world based on countries, and (2) also demonstrate a trend of the prevalence of lifetime and current e-cigarettes vaping.

RETRACTED

## Method

### Search strategy and selection of articles

This study was a systematic review and meta-analysis to determine the national, regional and global prevalence of e-cigarettes vaping. In this study, articles were searched in July 2020 without a time limit and only in articles published in English in Web of Science (ISI), Scopus, PubMed, and Ovid-MEDLINE. Contrary to what is mentioned in the protocol, we did not use Google Scholar to search for articles. Also, the reference sections of relevant systematic review articles were checked. In this study, the phrase of “lifetime prevalence” referred to e-cigarette vaping by a person during his/her lifetime, and the phrase of “current prevalence” referred to e-cigarette vaping during the last 12 months. The search strategy was performed with the keywords of “Electronic Cigarette” OR “Electronic Nicotine” OR “E-Cigarette” OR “Vaping” OR “E-Cig” (Additional file 1). This study was based on the PRISMA guideline (Fig. 1). The protocol of this study has been registered in the PROSPERO system (registration number: CRD42020183032).

**Fig. 1:** Flowchart of the systematic review process using PRISMA checklist

To select articles, first, all search results were entered into Endnote software and then reviewed by two authors separately and any disagreement was reviewed by the third author. At this stage, first, the titles and abstracts of the articles were reviewed, and if they were appropriate, they entered in the second stage of screening. In the second stage, the all articles were reviewed and articles that met the inclusion criteria were selected. The process of reviewing the selection of articles is shown in Fig. 1.

### Inclusion and exclusion criteria

Inclusion criteria included (1) papers published in English language, (2) cross-sectional, cohort, case–control, and intervention articles, (3) papers that reported the prevalence of e-cigarette vaping, and (4) papers that were published in full text. Exclusion criteria included qualitative papers, and papers that were published as review study, editorials comments, presentations or conference abstracts.

### Quality assessment

Methodological quality was assessed using the Joanna Briggs Institute’s critical appraisal tool [15] for prevalence studies. This tool evaluates the extent to which a study has addressed the potential biases in its design, conduct, and analysis. Studies were examined for representativeness, sample size, recruitment, description of study participants and setting, data coverage of the identified sample, reliability of the measured condition, statistical analysis, and confounding factors. Scores ranged from 0–9 with ≤ 5 as “low/moderate quality” and > 5 as “fair quality.” All studies selected for this meta-analysis were independently assessed by two authors (A.R. and A.J), and any disagreements between the two authors were reviewed and corrected by a third author.

RETRACTED

### Data extraction

All final papers entered into the study process were extracted from a pre-prepared checklist. The checklist included the surname of the first author, year of data collection, year of paper publication, target group, age of target group, place of study, type of study, the data gathering instrument, sample size, current and lifetime prevalence of e-cigarettes vaping, the prevalence of current e-cigarettes vaping in who had lifetime smoked conventional cigarettes, or currently smoking conventional cigarettes (Table S1). In this study, search, study selection, qualitative evaluation, and data extraction were conducted independently by two authors, and any disagreements between the two authors were reviewed and corrected by a third author.

### Data analysis

The pooled prevalence of e-cigarettes and a 95% confidence interval (CI) was calculated with raw data in STATA version 16 (Stata Corp LP, College Station, TX, USA). A random effects models (Der-Simonian Laird method) were used to combine data from individual studies. Q test and I2 statistic were used to calculate the heterogeneity between studies. I2 describes the percentage of total variation because of between-study heterogeneity [16]. Subgroup analysis was conducted according to the continent, study design, population study, and tools of assessment of e-cigarettes. Meta-regression was performed to explore the possible sources of heterogeneity. A *p*-value less than 0.05 was considered to be statistically significant.

## Results

In brief, a total of 146 eligible studies were identified and included in in the final analysis from 4026 potentially relevant articles with 5,495,495 participants. A flowchart of the inclusion and exclusion criteria of articles are shown in Fig. 1. The included studies were published between 2010 and 2020. The studies were conducted on four continents, with 67 studies in North America, 28 studies in Asia, 43 studies in Europe, and 8 studies in Australia/Oceania. Of the total studies included in this systematic review, 137 studies were cross-sectional and 9 studies were cohort studies (Table S1) [3–7, 12, 17–156].

### The prevalence of lifetime and current e-cigarettes vaping

The results of this study showed that the lifetime and current prevalence of e-cigarettes vaping were 23% (with a confidence interval (CI) of 95%: 21–25%) and 11% (95% CI: 10–11%), respectively (Fig. 2). The lifetime and current prevalence of e-cigarettes vaping among women were 16% (95% CI: 15–18%) and 8% (95% CI: 0.07–0.08%), respectively (Fig. 3). Also, the lifetime and current prevalence of e-cigarettes vaping among men were 22% (95% CI: 20–25%) and 12% (95% CI: 11–13%), respectively (Fig. 4).

RETRACTED

**Fig. 2:** Pooled lifetime and current prevalence of e-cigarettes vaping in all subjects

**Fig. 3:** Pooled lifetime and current prevalence of e-cigarettes vaping in women

**Fig. 4:** Pooled lifetime and current prevalence of e-cigarettes vaping in men

In this study, the lifetime prevalence of e-cigarettes vaping among adolescents and school students, adults, college students, and patients were 25% (95% CI: 21–30%), 19% (95% CI: 17–21%), 26% (95% CI: 15–37%), and 29% (95% CI: 16–43%), respectively (Fig. 5). Also, the current prevalence of e-cigarettes vaping in adolescent and school students, adults, college students, and patients were 11% (95% CI: 10–12%), 11% (95% CI: 10–12%), 14% (95% CI: 7–22%), and 10% (95% CI: 8–11%), respectively (Fig. 5). The lifetime and current prevalence of e-cigarettes by subgroups in women and men can be seen in Fig S1 and Fig S2.

**Fig. 5:** Pooled lifetime and current prevalence of e-cigarettes vaping in all subjects by study population, continent, type of study, and tools assessment

The lifetime prevalence of e-cigarettes vaping in the continents of America, Europe, Asia, and Oceania were 24% (95% CI: 21–27%), 26% (95% CI: 21–31%), 16% (95% CI: 11–20%), and 25% (95% CI: 18–33%), respectively (Fig. 5). The current prevalence of e-cigarettes vaping in the continents of America, Europe, Asia, and Oceania were 10% (95% CI: 9–10%), 14% (95% CI: 10–17%), 11% (95% CI: 10–11%), and 6% (95% CI: 4–8%), respectively (Fig. 5).

According to the type of study, the lifetime prevalence of e-cigarettes vaping in cohort studies and cross-sectional studies were 28% (95% CI: 11–45%) and 23% (95% CI: 21–25%), respectively (Fig. 5). Also, based on the type of study, the current prevalence of e-cigarettes vaping in cohort studies and cross-sectional studies were 13% (95% CI: 11–16%) and 11% (95% CI: 10–11%), respectively (Fig. 5).

In terms of assessment tools, the lifetime prevalence of e-cigarettes vaping in studies conducted by self-report and standard questionnaire were 23% (95% CI: 21–26%) and 20% (95% CI: 15–25%), respectively (Fig. 5). Also, in terms of assessment tools, the current prevalence of e-cigarettes vaping in studies conducted by self-report and the standard questionnaire were 12% (95% CI: 11–12%) and 5% (95% CI: 4–6%), respectively (Fig. 5). In this study, the current prevalence of e-cigarettes vaping in people who had lifetime used conventional cigarettes, and in current smokers (conventional cigarettes) were 39% (95% CI: 36–42%) and 43% (95% CI: 39–47%), respectively (Fig. 6).

RETRACTED

**Fig. 6:** Pooled current prevalence of e-cigarettes vaping in ex-smokers and current smokers

### The trend of current e-cigarettes vaping

The cumulative meta-analysis examined current e-cigarette vaping trends, which showed an upward trend from 2011 to 2014 and then a constant trend from 2014 to 2019 (Figure S3, Part A). The current prevalence of e-cigarettes among women first showed an upward and then a downward trends (Figure S4, part A). However, the current prevalence of e-cigarettes among men first showed an upward trend and then showed a constant trend (Fig S5, part A). The current prevalence of e-cigarettes vaping among adolescents and school students showed an upward trend. However, results of current e-cigarettes vaping among adolescents and school students showed an upward trend and among adults showed a downward trend (Fig S6, part A). The current prevalence of e-cigarettes vaping in continents of Americas and Asia first showed an upward trend and then showed an almost constant trend. The current prevalence of e-cigarettes vaping in Europe continent showed an upward trend (Fig S7, part A). The current prevalence of e-cigarettes vaping among people who had lifetime used conventional cigarettes and among current smokers (conventional cigarettes) first showed an upward trend and then showed an almost constant trend (Fig S8). The current prevalence of e-cigarettes vaping by subgroups among women and men can be seen in Fig S9 (part A) and Fig S10 (part A). The lifetime prevalence of e-cigarettes vaping by subgroups among women and men in each continent can be seen in Fig S11 (part A) and Fig S12 (part A).

### The trend of lifetime e-cigarettes vaping

The cumulative meta-analysis examined the lifetime e-cigarettes vaping, which showed an upward trend from 2011 to 2019 (Fig S3, part B). The trend of lifetime e-cigarettes vaping among women first showed an upward trend and then showed a constant trend (Fig S4, part B). Also, the trend of lifetime e-cigarettes vaping among men showed an upward trend and then showed a constant trend (Fig S5, part B). According to the results, the lifetime e-cigarettes vaping among adolescents and school students showed an upward trend (Fig S6, part B). The lifetime e-cigarettes vaping in the continents of the Americas, Asia, Europe, and Oceania showed an upward trend (Fig S7, part B). The lifetime prevalence of e-cigarettes vaping by subgroups among women and men can be seen in Fig S9 (part B) and Fig S10 (part B). The lifetime prevalence of e-cigarettes vaping by subgroups among women and men in every continent can be seen in Fig S11 (part B) and Fig S12 (part B).

RETRACTED

### Quality of included studies

The risk of bias and the quality of the included articles is illustrated in Table S2. All studies used an adequate sample size (100%) to determine the prevalence of e-cigarettes vaping. All studies (100%) used appropriate statistical analysis to measure the prevalence of e-cigarettes vaping. According to the Joanna Briggs Institute's Quality Assessment Checklist; the included articles had a score ranging from five to nine (Total nine-scored scale). Four studies scored nine out of nine (2.74%), fifty-seven studies scored seven to eight out of nine (39.04%) and the remaining eighty-five studies scored five to six out of nine score (58.22%) (Table S2) [3–7, 12, 17–156].

### Meta-regression analyses

Exploratory univariate meta-regression was conducted with the introduction of sample size, year of publication, tools of assessment, study design, continent, and population study for lifetime vaping and current vaping prevalence. The meta-regression coefficients for lifetime e-cigarettes vaping, 95% CI and *P*-value for these variables were, year of publication: β = 0.013, (95% CI: 0.0024, 0.0254, *p* = 0.01), sample size: β = -1.42e^−6^ (95% CI: -2.05e^−6^, -7.82e^−7^, *p* < 0.001), tools of assessment: β = -0.029, (95% CI: -0.098, 0.039, *p* = 0.39), continent: β = 0.010, (95% CI: -0.011, 0.032, *p* = 0.34), study design: β = -0.049, (95% CI: -0.170, 0.072, *p* = 0.42), study population: β = -0.0012, (95% CI: -0.028, 0.025, *p* = 0.92). The meta-regression coefficients for current e-cigarettes vaping showed that th95% CI and *P*-value for follow variables were, year of publication: β = 0.0065, (95% CI: 0.0037, 0.0092, *p* < 0.001), sample size: β = -1.88e^−6^ (95% CI: -2.30e^−6^, -1.46e^−7^, *p* < 0.001), tools of assessment: β = -0.059, (95% CI: -0.076, -0.043, *p* < 0.001), continent: β = 0.005, (95% CI: -0.0013, 0.010, *p* = 0.05), study design: β = -0.025, (95% CI: -0.042, -0.0075, *p* = 0.005), study population: β = 0.0037, (95% CI: -0.0022, 0.0097, *p* = 0.22).

## Discussion

This systematic review and meta-analysis study was conducted to determine the global prevalence of e-cigarettes vaping. In this study, the lifetime and current prevalence of e-cigarettes vaping in both sexes were 23% and 11%, respectively. The Europe continent had the high prevalence of e-cigarettes vaping and the lifetime and current of e-cigarettes vaping were 26 and 14 respectively. According to the results of this study, the overall trend of e-cigarettes vaping from 2011 to 2019 showed an upward trend. The current e-cigarettes vaping trend has been increasing from 2011 to 2014, and then there is a steady trend from 2014 to 2019.

RETRACTED

### Prevalence in men and women

The lifetime prevalence of e-cigarettes vaping among men and women were 22% and 16%, respectively. Also, the current prevalence of e-cigarettes vaping among men and women were 12% and 8%. In a study conducted in South Korea, the lifetime and current prevalence of e-cigarettes were 11.2% and 2% in men and 2.1% and 0.4% in women, respectively [117]. In a study conducted in Spain, the lifetime prevalence of e-cigarettes vaping among men and women were 8% and 5.3%, respectively [121]. The current prevalence of e-cigarettes vaping among Japanese men and women were 6.7% and 3.1%, respectively [136]. The lifetime prevalence of e-cigarettes vaping among Germany men and women were 9.2% and 6.7%, respectively, and the current prevalence of e-cigarettes vaping were 2.6% and 1.3%, respectively [115]. Among American men and women, the lifetime prevalence of e-cigarettes vaping were 9.6% and 7.4%, respectively, and current prevalence of e-cigarettes vaping were reported 2.6% and 2.1%, respectively [133]. Men and women use e-cigarettes for a variety of reasons. Men will start using e-cigarettes for reasons such as quitting smoking, health concerns related to conventional cigarette, and curiosity about e-cigarettes. In women, the recommendation to use e-cigarettes by family or friends is one of the important reasons for e-cigarettes vaping [157].

According to the results, the current prevalence of e-cigarettes among men first showed an upward trend and then showed a constant trend. Also, the current prevalence of e-cigarettes among women first showed an upward and then a downward trends. One of the reasons for the increasing trend of the current prevalence is the positive expectations of e-cigarettes including good taste, good social performance, and increased energy in men compared to women, while the only positive expectation of women to use e-cigarettes is weight loss due to e-cigarettes vaping [157]. The findings suggest that young women are more likely to use e-cigarettes, while pregnant women are less likely to use e-cigarettes due to the adverse effects of e-cigarettes [158]. The reason for the decrease of e-cigarettes vaping among women may be the failure of smoking consumption to help with weight loss and fitness. Also, women are generally more concerned about their health than men, and the reason for the reduced consumption may be due to greater awareness of the complications of e-cigarettes vaping.

### Prevalence in adolescent’s and school students

In this study, the lifetime and current prevalence of e-cigarettes vaping among adolescents and school students were 25% and 11%, respectively. In a study conducted in Russia, the lifetime and current prevalence of e-cigarettes vaping were 28.6% and 2.2%, respectively [114]. The current prevalence of e-cigarettes vaping among adolescents and school students is very wide in different countries, such as 1% in Mexico [159] and 9.9% in the United States [122]. In other countries such as China, the United Kingdom, Canada, and Poland, the current prevalence of e-cigarettes vaping were reported 1.2%, 2.2%, 3.6% and 3.5%, respectively [148, 150, 160]. According to the results, the trend of lifetime and current prevalence of e-cigarettes vaping in adolescents has been increasing, for example, the lifetime prevalence rate in the UK has increased from 22% in 2014 to 25% in 2016 [161], also the current prevalence rate in the United States has increased rapidly from 1.5% in 2011 to 20.8% in 2018 [162]. In various studies, a positive relationship has been found between the amounts of monthly allowance given by parents to their adolescent children, so as much as the amount of money is higher, the probability of e-cigarettes vaping is also higher by children [144, 163–165] and this factor could have been a reason to increase e-cigarettes vaping. Another reason for increasing the prevalence of e-cigarettes vaping could be the use of e-cigarettes to quitting conventional cigarette by adolescents. Therefore, this results indicate that families should pay more attention to their adolescent and children about e-cigarettes vaping. Also, as an important channel for e-cigarettes vaping education, health professionals could play an important role, especially for adolescents and school students. Additionally, banning the sale of e-cigarettes to people under 18 years may help reduce e-cigarettes vaping rates among adolescents and school students.

RETRACTED

### Prevalence in adults

In this study, the lifetime and current prevalence of e-cigarettes vaping among adults were 19% and 11%, respectively. In a study in South Korea, the lifetime and current prevalence of e-cigarettes were 6.6% and 1.1%, respectively [117]. In a study conducted in Spain, the lifetime prevalence of e-cigarettes vaping among adult men was 6.5% [121]. The current prevalence of e-cigarettes vaping in Japan has been reported to be 4.3% [136]. The current prevalence of e-cigarettes among adults varies from country to country, which can be influenced by various factors such as availability of these products and regulatory rules. For example, in China, the current prevalence of e-cigarettes vaping was 1.2%, while in the United States has been reported to be 5.5% [148, 159, 166]. However, the lack of laws on the sale of e-cigarettes and widespread access to tobacco in Chinese stores is a cause for concern about the increasing use of e-cigarettes, as in other countries [148]. In various studies conducted in different countries around the world, including Mexico, Australia, New Zealand, and Canada, the current prevalence of e-cigarettes has been reported to be 1.1%, 1.2%, 2.1%, and 2.9%, respectively [37, 167, 168]. Based on the results of this study, current prevalence of e-cigarettes vaping among adults showed decreasing trend. The downward trend in current prevalence may be due to increased awareness among adults about the harms and dangers of e-cigarettes, and the creation of regulatory laws that prohibit e-cigarette use.

### Prevalence in college students

In this study, the lifetime and current prevalence of e-cigarettes in college students were 26% and 14%. In a study conducted in five European countries including Slovakia, Belarus, Poland, Russia and Lithuania, the lifetime prevalence of e-cigarettes among college students were 34.4%, 42.7%, 45%, 33.4%, and 42.7%, respectively, and the current prevalence of e-cigarettes in these five countries were 2.3%, 2.7%, 2.8%, 4%, and 3.5%, respectively [2]. In a study conducted in the United States, the lifetime and current prevalence of e-cigarettes vaping among college students were 9% and 30%, respectively [130]. In another study among health science students in Saudi Arabia, the lifetime prevalence of e-cigarettes vaping has been reported to be 27.7% [137]. In a study conducted in Pakistan on medical students, the prevalence of e-cigarettes vaping was 13.9% [139], while in another study, the current prevalence of e-cigarettes vaping was 4.4% on medical students and 12.4% on non-medical students [2]. It has been reported that the reason for the low prevalence among medical students maybe their high awareness of the dangers of e-cigarettes vaping during the period of their education course [2]. The lifetime prevalence of e-cigarettes in Malaysian college students has been reported to be 20.4% [143]. Differences prevalence of e-cigarettes vaping in studies can be due to the different target groups, differences in age groups, and method of conducted the studies. According to the results of this study, the lifetime prevalence of e-cigarettes among college students showed increasing trend and the current prevalence of consumption has been decreasing. The reasons for the declining trend of the current prevalence of e-cigarettes can be cultural differences and the creation of laws to monitor and prohibit the use of e-cigarettes. Also, the prohibition of e-cigarettes vaping in the college can be effective in reducing e-cigarettes vaping.

RETRACTED

### Prevalence by continent

In this study, the lifetime prevalence of e-cigarettes vaping was 24% in the Americas, 26% in Europe, 16% in Asia and 25% in Oceania. Also, in this study the current prevalence of e-cigarettes vaping was 10% in the Americas, 14% in Europe, 11% in Asia, and 6% in Oceania. In a study conducted in 27 European countries, the lifetime prevalence of e-cigarettes increased from 7.2% in 2012 to 11.6% in 2016 [169]. One of the reasons for the increase in consumption in this continent may be because people usually use e-cigarettes to reduce or quit conventional cigarettes, but after a period of time, they start to use e-cigarettes continuously.

In this study, the lifetime prevalence of e-cigarettes vaping in the continents of Americas, Asia, Europe, and Oceania showed an upward trend. Also, the current e-cigarettes vaping in the continents of Americas and Asia first showed an upward trend and then showed an almost constant trend, but in Europe continent, it was showed an upward trend. In general, the use of e-cigarettes is increasing across different continents, possibly due to insufficient taxation of e-cigarettes. Also, given the increase in e-cigarettes in recent years, the law may not have been enacted yet. The reason for the differences in the prevalence of e-cigarettes in different continents may be due to the enactment of laws to reduce publicity, ban sales, increase taxes and conduct information campaigns in the field.

### Prevalence of e-cigarettes vaping among ex-smokers and current smokers

In this study, the current prevalence of e-cigarettes vaping in people who had lifetime used conventional cigarettes, and among current smokers were 39% and 43%, respectively. In a study conducted in Malaysia, the current prevalence of e-cigarettes vaping in who had lifetime smoked conventional cigarettes, and in current smokers conventional cigarettes were 4.3% and 8%, respectively [146]. In a study in the USA, the current prevalence of e-cigarettes vaping among current smokers has been reported to be 24.1% [128]. One of the reasons for e-cigarettes vaping among current smoker’s conventional cigarettes is the curiosity to try it, helping to quit and reduce conventional cigarette smoking. In a study conducted in Serbia, 12.8% of respondents reported that e-cigarettes vaping helped reduce their conventional cigarette smoking [153].

The current prevalence of e-cigarettes among people who had lifetime smoked conventional cigarettes or among current smokers first showed an upward trend and then t showed an almost constant trend. The reason for the increasing trend of e-cigarettes vaping may be the tendency of more smokers to quit or reduce conventional cigarettes, which can also be seen as both a threat and an opportunity. The threat aspect of this approach may be that a greater tendency to use e-cigarettes can lead to addiction to e-cigarettes. The opportunity aspect of this approach is that since most people have a tendency to quit smoking, e-cigarette can be a good option for quit or reducing conventional cigarettes.

RETRACTED

## Conclusion

According to the results of this study, it can be concluded that the prevalence of e-cigarettes is increasing worldwide. Therefore, it is necessary for countries to have more control over the consumption and distribution of e-cigarettes, as well as to formulate laws prohibiting the consumption of e-cigarettes in public places. Due to the increase in the prevalence of e-cigarettes among adolescents and school students, it is necessary that parents pay more attention to their children and also schools should also design and implement various educational programs to increase the awareness of adolescents and school students in this field. A broad program of behavioral, communications, and educational research is crucial to assess how youth perceive e-cigarettes and associated marketing messages, and to determine what kinds of tobacco control communication strategies and channels are most effective.

Besides, due to the high prevalence of e-cigarettes among current smokers, to quit or reduce their conventional cigarette smoking, more evidence is require in this regard and Clinical trial studies are also recommended to evaluate the benefits and harms of e-cigarettes vaping. The increase in e-cigarettes consumption in continental Europe compared to other continents indicates more detailed studies to identify the use of e-cigarettes, survey, and enact laws to ban e-cigarettes in this continent.

### Limitations and strengths

This study also had its limitations. Due to the use of studies whose data are collected through self-reporting data, the results of the study may be distorted due to measurement errors such as reporting bias and reminder bias. This self-reporting can lead to the misclassification of people that applies to smoke behavior in women, who are often underreported. Another limitation of this study was that due to the smaller number of studies that reported the lifetime prevalence of e-cigarettes vaping in pregnant women (2 studies) than the studies that reported the current prevalence of e-cigarettes vaping in this group (3 studies), the lifetime prevalence rate was lower than the current prevalence rate. One of the strengths of the study is that it includes cross-sectional, cohort, case–control, and intervention studies, and examines the prevalence of e-cigarettes in worldwide, and examines both the lifetime and current prevalence of e-cigarettes. It has also examined the prevalence of e-cigarettes in different subgroups including men, women, adults, adolescents, university students, by continents, and conventional cigarette users.

RETRACTED

## Supplementary Information

**Additional file 1. **Search Strategy.

**Additional file 2: Table S1.** Population characteristics of the studies reported the lifetime and current prevalence of electronic cigarette (e-cigarettes) vaping among women and men.

**Additional file 3: Table S2.** Qualities of studies included in the systematic review and meta-analysis.

**Additional file 4: Fig S1.** Pooled lifetime and current prevalence of e-cigarettes vaping by subgroups in women.

**Additional file 5: Fig S2.** Pooled lifetime and current prevalence of e-cigarettes vaping by subgroups in men.

**Additional file 6: Fig S3.** Cumulative meta-analysis of lifetime and current prevalence of e-cigarettes vaping in all subjects.

**Additional file 7: Fig S4.** Cumulative meta-analysis of lifetime and current prevalence of e-cigarettes smoking among women.

**Additional file 8: Fig S5.** Cumulative meta-analysis of lifetime and current prevalence of e-cigarettes vaping among men.

**Additional file 9: Fig S6.** Cumulative meta-analysis of lifetime and current prevalence of e-cigarettes vaping by study population.

**Additional file 10: Fig S7.** Cumulative meta-analysis of lifetime and current prevalence of e-cigarettes vaping by continent.

**Additional file 11: Fig S8.** Cumulative meta-analysis of current prevalence of e-cigarettes vaping in ex-smokers and current smokers. Pooled lifetime and current prevalence of e-cigarettes vaping by subgroups in women.

**Additional file 12: Fig S9.** Cumulative meta-analysis of lifetime and current prevalence of e-cigarettes vaping by subgroups in women.

**Additional file 13: Fig S10.** Cumulative meta-analysis of lifetime and current prevalence of e-cigarettes vaping by subgroups in men.

**Additional file 14: Fig S11.** Cumulative meta-analysis of lifetime and current prevalence of e-cigarettes vaping by subgroups in women in every continent.

**Additional file 15: Fig S12.** Cumulative meta-analysis of lifetime and current prevalence of e-cigarettes vaping by subgroups in men in every continent.

## Data Availability

Not applicable.

## Abbreviation

E-cigarettes: Electronic cigarettes
